The article "Molecular investigation and genetic diversity of Pediculus and Pthirus lice in France" was retracted in 2025. Reason: lack of ethics approval or compliance.

# Molecular investigation and genetic diversity of *Pediculus* and *Pthirus* lice in France

**DOI:** 10.1186/s13071-020-04036-y

**Published:** 2020-04-07

**Authors:** Nadia Amanzougaghene, Oleg Mediannikov, Tran Duc Anh Ly, Philippe Gautret, Bernard Davoust, Florence Fenollar, Arezki Izri

**Affiliations:** 1 Aix Marseille Univ, IRD, AP-HM, SSA, VITROME, Marseille, France; 2 IHU-Méditerranée Infection, Marseille, France; 3 Aix Marseille Univ, IRD, AP-HM, MEPHI, Marseille, France; 4 Department of Parasitology-Mycology, AP-HP, Hôpital Avicenne, Bobigny, France; 5 UMR “Émergence des Pathologies Virales” (EPV, Aix-Marseille University-IRD, 190-Inserm 1207 EHESP-IHU Méditerranée Infection), Marseille, France

**Keywords:** *Pediculus* lice, Pubic lice, *Bartonella quintana*, *Coxiella burnetii*, *Acinetobacter*, France

## Abstract

**Background:**

Humans are parasitized by three types of lice: body, head and pubic lice. As their common names imply, each type colonizes a specific region of the body. The body louse is the only recognized disease vector. However, an increasing awareness of head lice as a vector has emerged recently whereas the status of pubic lice as a vector is not known since it has received little attention.

**Methods:**

Here, we assessed the occurrence of bacterial pathogens in 107 body lice, 33 head lice and 63 pubic lice from Marseille and Bobigny (France) using molecular methods.

**Results:**

Results show that all body lice samples belonged to the *cytb* Clade A whereas head lice samples belonged to Clades A and B. DNA of *Bartonella quintana* was detected in 7.5% of body lice samples and, for the first time to our knowledge, in 3.1% of pubic lice samples. *Coxiella burnetii*, which is not usually associated with transmission by louse, was detected in 3.7% of body lice samples and 3% of head lice samples. To the best of our knowledge, this is the first report of *C. burnetii* in *Pediculus* lice infesting humans in France. *Acinetobacter* DNA was detected in 21.5% of body lice samples, 6% of head lice samples and 9.5% of pubic lice samples. Five species were identified with *A. baumannii* being the most prevalent.

**Conclusions:**

Our study is the first to report the presence of *B. quintana* in pubic lice. This is also the first report of the presence of DNA of *C. burnetii* in body lice and head lice in France. Further efforts on the vectorial role of human lice are needed, most importantly the role of pubic lice as a disease vector should be further investigated.

## Background

Human lice belong to the insect order Phthiraptera, suborder Anoplura (sucking lice) [1]. They complete their entire life-cycle on the host where they feed strictly on the blood by piercing the skin with their mouthparts [2]. Two species of lice parasitise humans: *Pediculus humanus* (represented by two forms, the head louse *P. h. capitis* and the body louse *P. h. humanus*); and the pubic or crab louse, *Pthirus pubis*. Chimpanzees are infested with *Pediculus schaeffi*, New World monkeys with *Pediculus mjobergi*, while gorillas with *Pthirus gorilla* [3, 4].

*Pthirus pubis* is prevalent worldwide and is present in all categories of the population [5]. The pubic louse lives in the hair of pubic area, but can occasionally infest several hairy areas on an individual, such as under the armpits, in the beard or mustache, or on the eyebrows and eyelashes [5, 6]. It is sexually transmitted and has often been found in combination with sexually transmitted infections [5, 6]. Currently, it is not known whether pubic lice carry an agent of human disease under natural conditions [6, 7].

*Pediculus humanus* is found in two forms (head and body lice) which are now usually considered members of a single species as opposed to separate species. They are morphologically very similar, but ecologically distinct and have different feeding patterns [2]. Head louse is confined to the scalp and feed on human blood every 4–6 hours [2]. Body louse lives in clothing and moves onto the skin to feed less frequently, but takes more large blood meals than the head louse [2, 8]. Head lice infestation is prevalent worldwide, particularly in school-aged children, regardless of hygienic conditions, while body lice is restricted to precarious populations living in poor sanitary conditions, such as the homeless, prisoners and war refugees [8, 9].

Body louse is the main vector of the bacteria responsible for trench fever (caused by *Bartonella quintana*), epidemic typhus (caused by *Rickettsia prowazekii*), and relapsing fever (caused by *Borrelia recurrentis*) [9, 10]; it is also strongly suspected in the transmission of the agent of the plague, *Yersinia pestis* [11–13]. Furthermore, the potential role of the body louse as a vector for other pathogenic bacteria has also been suspected, such as *Rickettsia conorii*, *Rickettsia typhi*, *Rickettsia akari*, *Coxiella burnetii* and *Acinetobacter* spp. [14–17]. In recent years, based on the combined evidence of both epidemiological and laboratory studies, there has been an increasing recognition of head lice as disease vectors, shifting the old-established paradigm, which implicated only body lice as disease vectors [18–21]. Indeed, experimental infections showed that head lice are able to acquire, maintain and transmit *R. prowazekii* and *B. quintana* [19, 20]. Moreover, DNA of several pathogenic bacteria has been found in head lice belonging to different clades, such as, *B. quintana*, *B. recurrentis*, *Y. pestis*, *C. burnetii*, *Rickettsia aeschlimannii* and *Acinetobacter* spp. [12, 18, 22–25].

Unlike *P. pubis*, the phylogeny of *P. humanus* has been extensively studied. Indeed, based on mitochondrial genes, six clades were described referred as Clade A, D, B, F, C and E [3, 26, 27]. Head lice encompass all clades diversity, while body lice belong to clades A and D only [3]. Of these, Clade A is the most prevalent and distributed worldwide [3, 28]. Clade D is found in DR Congo, the Republic of Congo, Ethiopia and Zimbabwe [3, 22, 27]. Clade B is found in the Americas, Europe, Australia, Algeria, South Africa, Saudi Arabia and in Israel among the remains of head lice from Roman times [3, 28, 29]. Clade F has been recently described in lice collected in French Guiana, Argentina and Mexico [3]. Clade C includes head lice observed in Ethiopia, the Republic of Congo and in Asia (Nepal, Pakistan and Thailand) [3, 28]. Lastly, Clade E consists of head lice from Senegal and Mali and has also been identified in head lice from Nigerian refugees in Algeria and from migrant communities living in Bobigny, France [3, 18, 30, 31].

The aim of the present work was to study the genetic diversity of head, body and pubic lice collected in Marseille and Bobigny in France and to investigate the presence of louse-borne pathogens in those lice.

## Methods

### Louse sampling

Louse sampling was performed over a period ranging from June 2017 to August 2018 in two regions of France: Marseille and Bobigny. In Bobigny, a town located close to Paris, lice were collected from patients attending the Avicenne Hospital. In total, 63 pubic lice, 24 head lice, and 54 body lice were collected from six patients (Table 1). In Marseille, lice were collected from homeless people at one shelter in May 2017. In total, 9 head lice and 53 body lice were collected from four individuals. All the sampled individuals were thoroughly examined for the presence of the all three types of lice. All visible lice were carefully removed using forceps. All collected lice were preserved in 70% alcohol and then transported to our IHU-Méd

**Table 1:** Summary of the pathogens detected in *Pediculus* and *Pthirus* lice collected from infested individuals in Bobigny and Marseille, France

Patients	Town	Individuals information	Type of lice (*n*)			*N*	Clade of *Pediculus* lice	Detection of			
			Pubic	Head	Body			*B. quintana*	*C. burnetii*	*Acinetobacter*	*Psychrobacter*
Patient 1	Bobigny	Patient	10	0	0	10	–	0	0	1 (pubic)	0
Patient 2	Bobigny	Patient	45	0	0	45	–	2 (pubic)	0	3 (pubic)	1 (pubic)
Patient 3	Bobigny	Patient	8	0	0	8	–	0	0	2 (pubic)	3 (pubic)
Patient 4	Bobigny	Schoolchild	0	7	0	7	7 B	0	0	0	0
Patient 5	Bobigny	Patient	0	0	15	15	15 A	2 (body)	0	0	0
Patient 6	Bobigny	Patient	0	17	39	56	56 A	0	2 (body)	5 (body)	1 (body)
Patient 7	Marseille	Homeless	0	5	0	5	5 B	0	0	0	0
Patient 8	Marseille	Homeless	0	0	11	11	11 A	3 (body)	1 (body)	2 (body)	0
Patient 9	Marseille	Homeless	0	0	12	12	12 A	1 (body)	0	1 (body)	1 (body)
Patient 10	Marseille	Homeless	0	4	30	34	34 A	2 (body)	2 (1 body, 1 head)	17 (2 head, 15 body)	0
Total			63	33	107	203	128 A (91.4%), 12 B (8.6%)	10 (4.9%)	5 (2.5%)	31 (15.3%)	6 (2.9%)

*Abbreviations*: N, total number; head, head lice; body, body lice; pubic, pubic lice

### DNA extraction

Prior to DNA isolation and in order to eliminate external contaminants, each louse was washed in iterranée Infection laboratory in Marseille (France).10% sodium hypochlorite for 10 min, 70% ethanol for 5 min, and finally rinsed three times with distilled water and dried on sterile filter paper. Genomic DNA was extracted using the DNA extraction kit, QIAamp Tissue Kit (Qiagen, Courtaboeuf, France) with the EZ1 apparatus according to the manufacturer’s instructions and stored at 4 °C until use in PCR amplifications.

### Molecular detection of the presence of pathogen DNA

#### Screening of pathogen DNA by real-time quantitative PCR (qPCR)

Each DNA sample was tested for the presence of *Bartonella* spp., *Borrelia* spp., *Anaplasma* spp., *Rickettsia* spp., *Acinetobacter* spp., *R. prowazekii*, *Y. pestis*, *B. quintana* and *C. burnetii*, using previously reported specific primers and probes (Additional file 1: Table S1). qPCRs were performed using a CFX96 Real-Time system (Bio-Rad Laboratories, Foster City, CA, USA) with Roche LightCycler 480 Probes Master Mix PCR kit (Roche Applied Science, Mannheim, Germany) in accordance with the manufacturer’s instructions. Negative (PCR mix and sterile water) and positive controls (including DNA of each target bacterium) were included for each qPCR run.

#### Conventional PCR and sequencing

All samples that tested positive using *Acinetobacter* genus-specific primers were subjected to standard PCR targeting a portion of the RNA polymerase β subunit (*rpoB*) gene (zone1), using the primers and all conditions previously described (Additional file 1: Table S1).

PCR amplification was performed in a Peltier PTC-200 model thermal cycler (MJ Research Inc., Watertown, MA, USA) and the AmpliTaq Gold 360 PCR Master Mix kit (Life Technologies, Villebon sur Yvette, France) in accordance with the manufacturer’s instructions. Successful amplification was confirmed *via* gel electrophoresis and PCR products were sequenced using a Big Dye Terminator kit and an ABI PRISM 3130 Genetic Analyser (Applied BioSystems, Courtabeauf, France) according to the manufacturer’s protocol.

### Genotypic status of lice

#### Pediculus lice

To identify the mitochondrial clades of *Pediculus* lice, all DNA samples (33 head lice and 107 body lice) were analyzed using clade-specific qPCR assays that targeted a portion of the cytochrome *b* (*cytb*) gene as previously described [18]. For phylogenetic analysis, DNA samples of 40 lice (7 body lice and 33 head lice) were randomly selected and subjected to standard PCR targeting a 347-bp fragment of *cytb* gene as previously described [32].

#### Pubic lice

DNA samples of 12 pubic lice were randomly selected and subjected to standard PCR targeting a 854-bp fragment of the mitochondrial gene *cytochrome c oxidase subunit 1* (*cox*1) using the primers and conditions previously described [33].

All louse amplicons were prepared and sequenced using similar methods as described above for the *rpoB* of *Acinetobacter* spp. The sequences of primers and probes used for qPCRs and conventional PCRs in this study are given in Additional file 1: Table S1.

### Data analyses

#### Sequences analysis

The electropherograms for each gene were assembled and edited using ChromasPro software (version 1.7.7; Technelysium Pty Ltd., Tewantin, Australia). All sequences obtained were analyzed using BLAST (www.ncbi.nlm.nih.gov/blast/Blast.cgi) and compared with sequences in the GenBank database. For *P. humanus* sequences, unique haplotypes were identified using DnaSP software (version 5.10) [34], then compared and combined with the *cytb* haplotypes dataset that we have reported previously [3].

#### Phylogenetic analysis

Phylogenetic trees were inferred based on the maximum likelihood (ML) method and the best-fit models were chosen using the Modeltest (version 3.7) [35]. Tree reconstruction was performed using MEGA software (version 7.0) [36]. *Pediculus humanus* haplotype network was constructed with the median joining method of Bandelt available in NETWORK5.0 (www.fluxus-engineering.com/sharenet.htm) using equal weights for all mutations [37].

#### Nucleotide sequence accession numbers

The newly generated sequences were submitted to the GenBank database under the accession numbers MN635415-MN635427 (*Acinetobacter* spp.), MN635428-MN635431 (*Psychrobacter* spp.), MN635435-MN635446 (*P. pubis*) and MN635432-MN635434 (*P. humanus*).

## Results

This study included 63 pubic lice, 33 head lice, and 107 body lice collected from 10 individuals from two regions of France, Marseille and Bobigny. All *Pediculus* lice were tested by qPCR to determine their clade. Our results showed that 91.4% (128/140) of analyzed lice were Clade A and only 8.6% (12/140) were clade B. According to louse ecotypes, all body lice were clade A (107/107), while 63.6% (21/33) of head lice were clade A and the remaining 36.4% (12/33) were clade B. For phylogenetic analysis, a total of 40 sequences (7 body and 33 head lice) were analyzed and their alignment with the publicly available sequences revealed the existence of 5 haplotypes including 3 new haplotypes referred here to as A70, A71 and B40. The remaining two haplotypes possessed the widespread haplotype A5 of Clade A and haplotype B36 of Clade B (Table 2). These haplotypes, together with our previously established dataset of all available body and head lice sequences were used to construct a maximum-likelihood (ML) tree and a median-joining (MJ) network (Figs. 1, 2).

**Table 2:** Haplotype frequency of head and body lice identified from France (Bobigny and Marseille)

Haplotype	Head lice	Body lice	Total	GenBank ID
A5	19	7	26	KM579542
A70	1	0	1	MN635432
A71	1	0	1	MN635433
B36	10	0	10	KM579559
B40	2	0	2	MN635434
Total	33	7	40

**Fig. 1:** Maximum-likelihood (ML) phylogenetic tree showing the relationship of haplotypes identified in this study with other *P. humanus* haplotypes. Phylogenetic inference was conducted in MEGA 7 using the maximum likelihood method under HKY + I + G model with 500 bootstrap replicates. There was a total of 270 positions in the final dataset. The scale-bar represents a 5% nucleotide sequence divergence

**Fig. 2:** *Cytb* haplotype networks of human body and head lice. Each circle indicates a unique haplotype, and variations in circle size are proportional to haplotype frequencies. Pie colors and sizes in circles represent the continents and the number of their sequence for a haplotype. The length of the links between nodes is proportional to the number of mutations. The types of haplotypes identified in this study are underlined

For pubic louse, a total of 12 samples were sequenced for the *cox*1 gene and examined in combination with the seven pubic louse sequences available on GenBank. The ML phylogenetic tree showing the position of all these sequences is given in Fig. 3.

**Fig. 3:** Maximum-likelihood (ML) phylogenetic tree showing the relationship of *P. pubis* amplified in this study with all *P. pubis* sequences available on GenBank. Phylogenetic inference was conducted in MEGA 7 using the maximum likelihood method under HKY + G model with 500 bootstrap replicates. There was a total of 776 positions in the final dataset. The scale-bar represents a 2% nucleotide sequence divergence

qPCR screening of all lice for *Acinetobacter* spp. detected 37/203 (18.2%) positive lice collected from 7 out of 10 (70%) people. We succeeded in amplifying a fragment of the *rpoB* gene for all positive lice. Unexpectedly, a BLAST search showed that only 31/37 of these sequences belong to the genus *Acinetobacter*, whereas the remaining 6/37 sequences belong to the genus *Psychrobacter* (Table 1).

For *Acinetobacter* spp., five species were identified, sharing 99–100% identity with their corresponding species. These are *A. baumannii* (23/203; 11.3%), *A. guillouiae* (4/203; 2%), *A. junii* (1/203; 0.5%), *A. nosocomialis* (2/203; 1%) and *A. schindleri* (1/203; 0.5%). According to louse species, all *A. schindleri* and *A. junii* DNA were found in pubic lice, while all *A. nosocomialis* DNA were found in body lice. *Acinetobacter guillouiae* DNA were found in both pubic (3 positive) and body (1 positive) lice, while *A. baumannii* DNA were detected in all three species, with body lice the most infected (20 positive), followed by head lice (2 positives) and only one pubic louse was found positive (Table 3). The phylogenetic position of *Acinetobacter* species is shown in Fig. 4.

**Table 3:** Sequences of *Acinetobacter* spp. and *Psychrobacter* spp. amplified in this study targeting *rpoB* gene

Sequence type	Type of louse			Total	GenBank ID
	Pubic louse	Head louse	Body louse		
*A. baumannii* ALF1	0	2	11	13	MN635415
*A. baumannii* ALF2	0	0	2	2	MN635416
*A. baumannii* ALF3	0	0	2	2	MN635417
*A. baumannii* ALF4	0	0	1	1	MN635418
*A. baumannii* ALF5	0	0	1	1	MN635419
*A. baumannii* ALF6	0	0	1	1	MN635420
*A. baumannii* ALF7	1	0	0	1	MN635421
*A. baumannii* ALF8	0	0	2	2	MN635422
*A. guillouiae* ALF9	0	0	1	1	MN635423
*A. guillouiae* ALF10	3	0	0	3	MN635424
*A. junii* ALF11	1	0	0	1	MN635425
*A. nosocomialis* ALF12	0	0	2	2	MN635426
*A. schindleri* ALF13	1	0	0	1	MN635427
*Psychrobacter* sp. PLF14	1	0	0	1	MN635428
*Psychrobacter* sp. PLF15	2	0	0	2	MN635429
*Psychrobacter* sp. PLF16	1	0	0	1	MN635430
*Psychrobacter* sp. PLF17	0	0	2	2	MN635431
Total	10	2	25	37

**Fig. 4:** Phylogenetic tree highlighting the position of *Acinetobacter* spp. and *Psychrobacter* spp. identified in this study. Phylogenetic inference was conducted in MEGA 7 using the maximum likelihood method under TrN + G model with 500 bootstrap replicates. There was a total of 350 positions in the final dataset. The scale-bar represents a 10% nucleotide sequence divergence

For *Psychrobacter* species, BLAST analysis shows a homology identity score of less than 91% with *Psychrobacter* sequences available in the GenBank database. Furthermore, all the sequences obtained showed a homology identity of 80–86% to each other, which means that each of these sequences is likely to be a potential yet undescribed new species. In the phylogenetic tree (Fig. 2), the sequences of all these potential new species formed separate and well-supported branches, which clustered together within the clade that contains *Psychrobacter* species.

In 10 (4.9% of 203) lice (8 body lice and 2 pubic lice) infesting five people, we detected *B. quintana* DNA. Six positive body lice were collected from 3 homeless individuals from Marseille, while the two remaining positive body lice were from one patient from Bobigny. The two positive pubic lice were collected from one patient from Bobigny. None of the head lice were positive for *B. quintana* DNA. *Coxiella burnetii* DNA was detected in 5 (2.5% of 203) tested lice, one was detected in head lice and four detected in body lice. None of the pubic lice were positive for *C. burnetii* DNA (Table 1).

All bacterial qPCRs targeting *Borrelia* spp., *Anaplasma* spp.*, Rickettsia* spp., *Acinetobacter* spp., *R. prowazekii* and *Y. pestis* were negative.

## Discussion

In the present study, we report the molecular data on the *Pthirus* and *Pediculus* lice infesting French individuals from Marseille and Bobigny. To the best of our knowledge, this is the first study of its kind in France, which examines both *Pthirus* and *Pediculus* lice from the same people.

The analysis of 33 head lice and 107 body lice mitochondrial clades revealed the presence of two *cytb* clades, A and B, distributed through 5 haplotypes. The most prevalent clade was Clade A (91.4% of 140) comprising both body lice and head lice whereas all Clade B found (8.6% of 140) comprised head lice. Our finding corroborates the previous *Pediculus* lice studies showing the presence of these two clades in France [3, 26, 29, 30]. Moreover, our results support the idea that these two clades were the dominant lineage in this country. Previous studies have shown the presence of clades E and C in addition to these two clades [3, 30]. Our sampling did not encounter any new specimens of these two clades, possibly due to the reduced number of lice involved in this study.

Unlike *Pediculus* lice, the phylogenetic position of *Pthirus* lice never received substantial attention, as reflected by the low number of pubic louse sequences available in the GenBank database, only seven *cox*1 sequences were found. All these sequences were added to the 12 sequences obtained in our study and used to construct the phylogenetic tree (Fig. 3). Despite that the *cox*1 gene is a fast-evolving marker and among the most commonly used in louse phylogenetic studies [33], the tree produced was not informative, possibly due to the few numbers of the lice sequences examined. The present study revealed the need for more detailed studies on pubic lice from different countries targeting different molecular makers in order to better understand their genetic diversity and build a robust phylogeny of the relationship between pubic lice.

*Bartonella quintana* can cause trench fever, bacillary angiomatosis, endocarditis, chronic lymphadenopathy and chronic bacteremia [8]. Body lice are the main known vector, but the role of head lice as a vector has been the subject of much discussion and speculation in recent years [10, 18, 19, 21, 23–25]. *Bartonella quintana* infection is the most common re-emerging louse-borne disease among homeless people in cities in the USA and Europe [38–40]. Studies of homeless populations have reported a prevalence of 7–22% for body louse infestations and 2–30% for *B. quintana* infections [38]. The main predisposing factors of this infection include poverty and unhygienic living conditions [39]. In the present study, *B. quintana* DNA was detected in eight out of 107 body lice tested. Two of the positive body lice infested one patient from Bobigny. The other six positive body lice were infesting three homeless individuals from Marseille, confirming that homeless people are among the population groups most vulnerable to infestation by lice and their associated pathogens.

Interestingly, two pubic lice infesting one patient from Bobigny were also found positive to *B. quintana* DNA. To the best of our knowledge, this is the first report of the presence of *B. quintana* in pubic lice. Although there is no available information on the infection status of the sampled individual, it is important to know that, as in the case of *Pediculus* lice, *Pthirus* lice are blood-feeding insects, which are predisposed to uptake any blood microorganisms while feeding on their human host. Theoretically, it is feasible that they can transmit any of these agents, being ingested with blood meal if they are capable of surviving in the insect’s midgut. Follow-up experiments are needed to investigate the potential role of pubic lice in the transmission of *B. quintana*.

*Coxiella burnetii* is the agent of Q fever, a globally widespread zoonosis that infects a wide range of animals, from arthropods to humans [41]. Infection in humans typically occurs through inhalation of contaminated aerosols or ingestion of infected animal products [41, 42]. Ticks have also been implicated as vectors [42]. Although human lice are not a known vector of *C. burnetii*, several reports suggest that they may play a role, under favorable epidemiological circumstances, in its transmission to humans [18, 43]. Indeed, under experimental conditions, it is possible to infect body lice with *C. burnetii* [43]. Moreover, a field study in Rwanda showed that body lice recovered from an area where an epidemic of Q fever occurred three months previously, are capable of transmitting *C. burnetii* to Guinea pigs [14, 43]. Furthermore, in recent studies, *C. burnetii* DNA was detected in 10.5% of 524 body lice infesting homeless individuals in Algeria, in 1% of 600 head lice from Mali and in 8.1% of 37 Nigerian refugees arriving in Algeria [18, 31, 44]. In the present study, the DNA of *C. burnetii* was detected in both head lice (3%, *n* = 33) and body lice (3.7%, *n* = 107) infesting 30% of the 10 people studied. Two of the five positive lice were from a patient living in Bobigny and the remaining three positive lice were from two homeless people living in Marseille. To our knowledge, this is the first report of the presence of *C. burnetii* DNA in head and body lice infesting individuals in France. Our results reinforce findings from previous studies that head and body lice may act as vectors of *C. burnetii*, which warrants further investigation.

In this study, we also assessed the collected lice for the presence of *Acinetobacter* species. More attention is now being paid to the reservoirs of these ubiquitous opportunistic pathogens, particularly to *A. baumannii*, which is known to be a major cause of nosocomial infections in humans, due to the increasing incidence of antibiotic-resistant treatment worldwide [45]. In total, DNA of *Acinetobacter* was detected in 23 body lice, two head lice, and six pubic lice. Five species were identified among with *A. baumannii* was the most prevalent (11.3%), followed by *A. guillouiae*, *A. nosocomialis*, *A. junii* and *A. schindleri*.

Body lice were found to be positive for DNA of three species of *Acinetobacter*, with *A. baumannii* being the most prevalent (86.9%), followed by *A. nosocomialis* (8.7%) and *A. guillouiae* (4.3%). This is consistent with previous reports showing that *A. baumannii* is the most abundant species found in body lice, as shown by its detection in 21% of body lice collected worldwide [46] and in 100% of body lice from Bobigny [30]. Regarding head lice only, *A. baumannii* was detected, which may be due to the fact that only a small number of head lice were analyzed. In previous studies, DNA of several *Acinetobacter* has been detected within head lice including: *A. junii*, *A. ursingii*, *A. johnsonii*, *A. schandleri*, *A. lwoffii*, *A. nosocomialis*, *A. towneri*, *A. schindleri*, *A. radioresistens*, *A. calcoaceticus* and *A. variabilis* [22, 30, 31, 47]. The following four species were found in pubic lice: *A. baumannii*, *A. guillouiae*, *A. junii* and *A. schindleri*. To our knowledge, this is the first report of DNA of these *Acinetobacter* species in being detected in pubic louse. To date, there is only one study in which *A. johnsonii* DNA was detected in four of eight pubic lice collected in Algeria [47].

Currently, despite the fact that several studies have demonstrated widespread infection of lice with several species of *Acinetobacter* [48], the association between *Acinetobacter* and human lice is still poorly understood. In an investigation conducted by Vallenet et al. [49], it was found that the genome of *A. baumannii*-SDF body louse strain had several hundred insertion sequence elements which have played a crucial role in reducing its genome compared to the human multidrug-resistant *A. baumannii* AYE strain, and whose catabolic capacities were low. Their finding suggests the specific adaptation of this strain to the louse environment niche [49], indicating that lice may constitute a natural reservoir of *Acinetobacter.* Moreover, it is still unknown how these lice acquire and transmit *Acinetobacter* infections to their human hosts. Several reports have suggested that the infection could occur after the ingestion of an infected blood meal from infected individuals [16, 46, 50]. Indeed, an experimental study demonstrated that the body louse, feeding on bacteremic rabbits, is able to acquire and maintain a persistent life-long infection with *A. baumannii* and *A. lwoffii* and disseminate viable organisms in their feces [16]. However, in a recent study conducted on homeless individuals to assess the presence of *A. baumannii* DNA on human skin, blood and in body lice collected from the same individuals, the authors found a strong association between body lice infestation and *A. baumannii* DNA skin-carriage, while all blood cultures and real-time PCR on blood samples were negative for *A. baumannii* [51]. They concluded that body lice probably become infected with *A. baumannii* while biting through the colonized skin and then likely transmit the bacteria in their feces [51]. Obviously, more effort is needed to study the specifics of the associations between human hosts, lice and *Acinetobacter* infections.

## Conclusions

Herein we report molecular data in both *Pthirus* and *Pediculus* lice from France. Polygenetic analysis of *Pediculus* lice confirmed that head and body lice from France belong to Clades A and B, as reported by others. Several *Acinetobacter* species were detected in both *Pediculus* and *Pthirus* lice, reinforcing the hypothesis that these lice may be a preferential host for these bacteria. Furthermore, we detected the presence of *C. burnetii* in both body and head lice which is not usually associated with louse transmission, suggesting that these lice may act as the vectors of other pathogenic bacteria, beside three classically recognized louse-borne pathogenic bacteria, i.e. *B. recurrentis*, *R. prowazekii* and *B. quintana*. Taken together, our results suggest that there is still much to learn about human lice and their associated pathogens. Moreover, to the best of our knowledge, our results report for the first time the presence of *B. quintana* DNA in pubic lice, taking into account that the role of pubic lice in the transmission of pathogens has never received substantial attention to date, which is an area of interest for future studies.

## Supplementary information

**Additional file 1: Table S1.** Oligonucleotide sequences of primers and probes used for real-time PCR and conventional PCR in the present study.

## Data Availability

All data generated or analyzed during this study are included in this published article and its additional file. The newly generated sequences were submitted to the GenBank database under the accession numbers MN635415-MN635427 (*Acinetobacter* spp.), MN635428-MN635431 (*Psychrobacter* spp.), MN635435-MN635446 (*P. pubis*) and MN635432-MN635434 (*P. humanus*).

## Abbreviations

qPCR: Real-time quantitative PCR
PCR: Polymerase chain reaction
*Cytb*: Cytochrome *b*
*cox*1: Cytochrome *c* oxidase subunit 1
*rpoB*: RNA polymerase β subunit
ML: Maximum likelihood
MJ: Median joining
